RETRACTED

# Mesenchymal stem cell-derived exosomal miR-146a reverses diabetic β-cell dedifferentiation

**DOI:** 10.1186/s13287-021-02371-0

**Published:** 2021-08-11

**Authors:** Qin He, Jia Song, Chen Cui, Jinbang Wang, Huiqing Hu, Xinghong Guo, Mengmeng Yang, Lingshu Wang, Fei Yan, Kai Liang, Zhaojian Liu, Fuqiang Liu, Zheng Sun, Ming Dong, Xinguo Hou, Li Chen

**Affiliations:** 1 Department of Endocrinology, Qilu Hospital, Cheeloo College of Medicine, Shandong University, No. 107 Wenhua Xi Road, Jinan, 250012 Shandong China; 2 Department of Cell Biology, Cheeloo College of Medicine, Shandong University, Jinan, 250012 China; 3 Institute of Endocrine and Metabolic Diseases of Shandong University, Jinan, 250012 China; 4 Key Laboratory of Endocrine and Metabolic Diseases, Shandong Province Medicine & Health, Jinan, 250012 China; 5 Jinan Clinical Research Center for Endocrine and Metabolic Diseases, Jinan, 250012 China

**Keywords:** Exosome, Mesenchymal stem cell, Type 2 diabetes mellitus, β-cell dedifferentiation, miR-146a

## Abstract

**Background:**

Mesenchymal stem cells (MSCs) show promising therapeutic potential in treating type 2 diabetes mellitus (T2DM) in clinical studies. Accumulating evidence has suggested that the therapeutic effects of MSCs are not due to their direct differentiation into functional β-cells but are instead mediated by their paracrine functions. Among them, exosomes, nano-sized extracellular vesicles, are important substances that exert paracrine functions. However, the underlying mechanisms of exosomes in ameliorating T2DM remain largely unknown.

**Methods:**

Bone marrow mesenchymal stem cell (bmMSC)-derived exosomes (bmMDEs) were administrated to T2DM rats and high-glucose-treated primary islets in order to detect their effects on β-cell dedifferentiation. Differential miRNAs were then screened via miRNA sequencing, and miR-146a was isolated after functional verification. TargetScan, reporter gene detection, insulin secretion assays, and qPCR validation were used to predict downstream target genes and involved signaling pathways of miR-146a.

**Results:**

Our results showed that bmMDEs reversed diabetic β-cell dedifferentiation and improved β-cell insulin secretion both in vitro and in vivo. Results of miRNA sequencing in bmMDEs and subsequent functional screening demonstrated that miR-146a, a highly conserved miRNA, improved β-cell function. We further found that miR-146a directly targeted *Numb*, a membrane-bound protein involved in cell fate determination, leading to activation of β-catenin signaling in β-cells. Exosomes derived from miR-146a-knockdown bmMSCs lost the ability to improve β-cell function.

**Conclusions:**

These findings demonstrate that bmMSC-derived exosomal miR-146a protects against diabetic β-cell dysfunction by acting on the NUMB/β-catenin signaling pathway, which may represent a novel therapeutic strategy for T2DM.

RETRACTED

**Supplementary Information:**

The online version contains supplementary material available at 10.1186/s13287-021-02371-0.

## Background

Type 2 diabetes mellitus (T2DM) is characterized by insufficient β-cell mass and insulin resistance and has become a worldwide disease due to its increasing morbidity [1]. This T2DM-induced decline in β-cell mass is attributed to a decrease in both β-cell number and function [2]. It has been suggested that reduced β-cell mass is the result of apoptosis [3]. However, recent data challenge the β-cell apoptosis hypothesis. These data indicate that dedifferentiation represents an alternative mechanism explaining the loss of functional β-cell [4, 5]. Dedifferentiated β-cells lose their insulin secretion capacity and transform into endocrine progenitor cells with multi-directional differentiation potential, characterized by the re-expression of Ngn3, thereby causing the total amount of functional β-cells to decline [6, 7]. Interventions of β-cell dedifferentiation can reverse hyperglycemic phenotypes and slow the progression of diabetes. Therefore, safe and effective treatments that reverse β-cell dedifferentiation may represent novel and promising therapeutic strategies for T2DM.

Recently, mesenchymal stem cell (MSC)-based therapy has offered a promising strategy for treating diabetes. Some clinical studies have found that MSCs and their derivatives can significantly improve fasting blood glucose, C-peptide levels, HbA1c levels, and insulin secretion [8–10], with no significant side effects having yet been observed. Among MSCs, bone marrow MSCs (bmMSCs) have shown significant effects in regulating β-cell mass and in ameliorating chronic high-glucose-induced β-cell injury [11, 12]. Our previous research has also confirmed that bmMSCs can improve diabetic islet microcirculation via Wnt4-β-catenin signaling [13]. Although these studies have documented improved β-cell function after MSC infusion, whether decreased β-cell dedifferentiation is involved in improved β-cell mass and insulin secretion has received less intention. In the present study, we directly address this question.

Exosomes are extracellular nanoparticles with lipid-bilayer membranes [14]. Exosomes can directly deliver effectors—such as proteins, mRNAs, and microRNAs—from secretory cells to recipient cells [15, 16]. MSCs can secrete larger amounts of exosomes compared to those of terminally differentiated cells [17]. MSC-derived exosomes can reverse peripheral insulin resistance and relieve cellular destruction [18, 19]. Compared to MSCs, exosomes have lower immunogenicity and lower risk of aneuploidy and can be more easily mass-produced, all of which make them more attractive therapeutic agents. MicroRNAs are small, non-coding RNAs that exert many biological roles by negatively regulating mRNA expression at the post-transcriptional level [20]. Recent studies have demonstrated that specific miRNAs play a vital role in regulating β-cell activities and are also involved in the development of diabetic vascular complications [21]. However, it is unknown whether bmMSC-derived exosomal miRNAs affect β-cell dedifferentiation.

RETRACTED

To elucidate the effects of bmMSCs on β cells, in the present study, we first demonstrated that bmMSC-derived exosomes (bmMDEs) reversed β-cell dedifferentiation and ameliorated β-cell function both in vitro and in vivo. miRNA sequencing was then used to further explore the role of bmMDEs. Finally, we showed that beneficial effects of bmMDEs on β-cell dedifferentiation were mainly achieved via the miR-146a-5p/*Numb*/β-catenin pathway. Taken together, our findings shed light on the potential of an MSC-derived exosome-based therapeutic approach for treating diabetes.

## Methods

### Cell culture and treatments

Rat primary bmMSCs were isolated as previously described [22]. Briefly, femurs and tibiae were obtained from Sprague-Dawley rats after euthanasia via an anesthetic overdose. The bone marrow was harvested by flushing the cavities of rats with DMEM/F12 medium (Gibco, Invitrogen, Carlsbad, CA) supplemented with 20% fetal bovine serum (FBS, depletion of exosomes by ultracentrifugation; Gibco). The media were changed after 24 h, and cells were at approximately 80% confluency when they were passaged. DMEM/F12 with 10% FBS was used in the subsequent cultures. The third to fourth generations of cells were used for experiments.

The INS-1 cell line was obtained from Nanjing Medical University, PR China. Cells were cultured in the RPMI-1640 medium (Gibco) supplemented with 15% FBS (depletion of exosomes by ultracentrifugation), 10 mM of Hepes (Sigma-Aldrich, St. Louis, MO), 1 mM of sodium pyruvate (Sigma-Aldrich), 2 mM of L-glutamine (Gibco), and 50 μmol/L of β-mercaptoethanol (Sigma-Aldrich) at 37°C with 5% CO_2_. Cells were inoculated in a six-well plate and were cultured in a medium containing 11.1 mmol/L (control) or 35 mmol/L of glucose (high glucose, HG) for 72 h with or without INS-1 cell-derived exosomes (IDEs, 30 μg/mL, normal control exosomes) or bmMDEs (30 μg/mL). Mannitol (MA, 35 mmol/L, SM8120, Solarbio) was used as an osmotic pressure control.

### Isolation and characterization of exosomes

Isolation and purification of exosomes were performed according to standard methods as described previously [23]. Briefly, the bmMSC culture medium was collected after being replaced with an exosome-free medium for 48 h. The conditioned medium was centrifuged at 300*g* for 10 min and was then centrifuged a second time at 2000*g* for 20 min to remove cells and apoptotic bodies. Next, samples were centrifuged at 10,000*g* for 30 min and were then filtered through a 0.22-μm filter to remove cellular debris. The final supernatant was centrifuged at 120,000*g* for 70 min at 4°C to pellet exosomes. Ultracentrifugation experiments were performed with an Optima MAX-XP (Beckman Coulter, USA). All of the exosome-containing pellets were resuspended in PBS or were lysed in RNA lysis buffer for further analysis. Exosomes were observed using a transmission electron microscope (TEM; JEM-1400, JEOL, Japan) and were quantified by a Nano-Sight NS300 (Malvern Instruments Ltd, UK).

RETRACTED

### Tracing of exosomes in INS-1 cells

Exosomes were labeled with a PKH67 Green Fluorescent Cell Linker Kit (PKH67, Sigma-Aldrich) according to the manufacturer’s protocol. First, 1 mL of Diluent C was added to the exosomes diluted in PBS. Then, 4 μL of PKH67 dye was added to 1 mL of Diluent C and was then incubated with exosomes (protected from light) for 4 min. To bind excess dye, 2 mL of 1% BSA was added to the reaction system. Re-extraction of labeled exosomes was performed by ultracentrifugation and subsequent dilution in 100 μL of PBS. The labeled exosomes were incubated with INS-1 cells. Fluorescence signals were detected by an Olympus BX53 fluorescent microscope.

### Animals and diets

Four-week-old male Sprague-Dawley rats (60–70 g) were purchased from Synergy Pharmaceutical Bioengineering Co., Ltd (Nanjing, China, Ethical number: DWLL-2015-005). After 1–2 weeks of adaptive feeding, the rats were given a 45% high-fat diet (HFD) for 4 weeks, whereas the control group rats were fed with a normal chow diet. These HFD rats were then injected intraperitoneally with STZ (30 mg/kg in 0.1 M citrate-buffered saline, pH=4.5, single dose, S0130; Sigma-Aldrich) after fasting for 12 h. T2DM rats were identified as having fasting glucose ≥ 16.7 mmol/L. STZ-treated rats continue HFD for another 13 weeks. All animal experimental protocols were approved by the Animal Ethics Committee of Shandong University.

### Treatment with bmMDEs in T2DM rats

T2DM rats were divided into the following five groups (*n* = 7/group): PBS, bmMSCs, bmMDEs, bmMDEs^miR-NC KD^, and bmMDEs^miR-146a KD^. bmMSCs (5×10^6^ cells/rat) were suspended in PBS and injected via the tail vein every 2 weeks for five cycles after STZ injections. Exosomes (10 mg/kg) were injected into rats via the tail vein every 3 days for 10 weeks. The normal control group (control, *n*=7) was injected intravenously with an equal volume of PBS (Fig. S7 for a more detailed experimental procedure). For exosome-tracking in vivo, Cy7-labeled exosomes were delivered into T2DM rats via tail-vein injections, and each rat and its harvested organs were imaged using an IVIS200 imaging system (Xenogen Corp., Alameda, CA, USA) at 24 h after injection. During the experiments, no animals became severely ill or died. All animal experimental protocols were approved by the Animal Ethics Committee of Shandong University.

RETRACTED

### Analysis of metabolic parameters

Rats were fasted for 3 h before measuring blood glucose levels. Body weight (BW) and food intake were monitored weekly. Intraperitoneal glucose tolerance tests (IPGTTs) and intraperitoneal insulin tolerant tests (IPITTs) were performed after the last intervention. IPGTTs were performed following overnight fasting. Blood glucose levels were detected at 0, 30, 60, 120, and 180 min after intraperitoneal injections of glucose (1.5 g/kg, Sigma-Aldrich). For IPITTs, rats were provided free access to food and water. Blood glucose levels were measured at 0, 30, 60, 120, and 180 min after intraperitoneal injections of insulin (2 IU/kg, Wanbang Pharmaceutical, Jiangsu, China).

### Isolation and intervention of islets from rats

Pancreatic tissues from rats were isolated after anesthesia. A syringe was pumped with 1 mg/mL of Collagenase V (C9263; Sigma-Aldrich) and was then replaced with a fine syringe needle inserted into the pancreas. The outflow of the enzymatic solution was re-injected 2–3 times. The harvested pancreas was then placed into a digestive bottle, and it was then digested at 37°C for 15 min. Subsequently, the sample was removed from the water bath and was lightly shaken 12 times. Ice-cold Hanks solution (with calcium and magnesium) was added to the digestive bottle and was shaken to stop collagenase digestion, after which the sample was placed on ice three times. Finally, the clean islets were hand-picked under a stereoscopic microscope. After preincubation overnight, the islets from Sprague-Dawley rats were exposed to 5.0 mmol/L (control) or 35 mmol/L of glucose (high glucose, HG) with or without IDEs (30 μg/mL) or bmMDEs (30 μg/mL) for 72 h. The islets from control, T2DM, and T2DM + bmMDE rats were pre-cultured overnight, after which they directly proceeded to the next experiment. MA (35 mmol/L) was used as an osmotic pressure control.

### Glucose-stimulated insulin secretion (GSIS)

After the corresponding intervention was completed, glucose-starved INS-1 cells and islets (50–60 islets in each group) were assessed in Krebs–Ringer bicarbonate solution (KRBS) containing 2.5 mmol/L of glucose at 37°C for 1 h. The supernatant was collected before being incubated in KRBS containing 25 mmol/L of glucose for another 1 h at 37°C. The supernatant was collected and insulin levels were detected using a commercial kit (Blue Gene, Shanghai, China) to evaluate stimulated insulin release. The final insulin content was normalized to the protein concentrations of cells and islets.

RETRACTED

### Immunofluorescence staining

INS-1 cells and paraffin sections of pancreatic tissue were incubated with the following antibodies: insulin (ab7842; Abcam), glucagon (ab10988; Abcam), PDX1 (5679; Cell Signaling Technology), FOXO1 (2880; Cell Signaling Technology), neurogenin3 (NGN3, sc-3744042; Santa Cruz, USA), OCT4 (GTX101497; GeneTex, CA, USA), and NUMB. After incubated with the fluorescence-conjugated secondary antibodies, the cell nuclei were stained with DAPI. Digital images were captured using an Olympus BX53 fluorescence microscope. Immunofluorescence staining statistics are measured from 3 to 5 rats per group, or 4–5 pancreas sections per rat for 15–20 islets. Quantitative analysis was performed using the CytoNuclear count function of the Image Pro-Plus software. Mean β-cell percentage per islet = average (β-cell number/total islet cell number) × 100%. Densitometry of staining was performed using ImageJ. Images were separated by color and inverted to black and white, and the integrated density was calculated for each stain using the tracing function.

### Real-time quantitative PCR (RT-qPCR)

Total RNAs were extracted from INS-1 cells and islets using MicroElute Total RNA Kit (Omega Bio-Tek, Doraville, GA, USA). Total miRNAs were extracted by a miRcute miRNA isolation kit (TIANGEN Biotech, Beijing, China) according to the manufacturer’s instructions. The sequences of above primers are listed in Supplementary Table 1. Real-time PCR was conducted with the SYBR Green PCR kit (catalog no. RR820B; Takara), and quantification was achieved by normalization using β-actin or U6 as the control.

### Small RNA library construction and sequencing

Total RNA was extracted using Trizol reagent (Invitrogen, CA, USA) following the manufacturer’s procedure. The total RNA quantity and purity were analyzed with a Bioanalyzer 2100 and an RNA 6000 Nano LabChip Kit (Agilent, CA, USA) with RIN number >7.0. Approximately 1 μg of total RNA was used to prepare a small RNA library according to the protocol of TruSeqTM Small RNA Sample Prep Kits (Illumina, San Diego, USA). Additionally, single-end sequencing (36 bp) was performed on an Illumina Hiseq2500 Lianchuan Biotechnology (LC-BIO, Hangzhou, China) following the vendor’s recommended protocol.

RETRACTED

### Luciferase reporter assay

To identify the binding site between miR-146a and *Numb*, INS-1 cells were transfected with a luciferase construct containing *Numb* with the wild-type or a mutated version of the binding site and then co-transfected with miR-NC or miR-146a mimics (GenePharma, Shanghai, China). Luciferase activities were detected after 48 h of transfection by using a Dual-Luciferase kit (Promega, Madison, USA) according to the manufacturer’s instructions.

### RNA interference and plasmids

siRNAs (siNC, siNUMB), plasmid vectors (vector containing *Numb* and empty vector), mimics/inhibitors of indicated miRNAs, and lentiviral vectors (vectors containing miR-146a sponge inhibitor and control) were prepared by GenePharma (Shanghai, China). The target sequence of Rattus-*Numb* (NM_133287.1) was 1799 bp, the vector was pcDNA3.1(+), and the restriction site was NheI-NotI. The sequences of siRNAs and miRNA mimics/inhibitors referred above are listed in the Supporting Information, namely in Tables S1 and S2.

### Statistical analysis

Three independent experiments were performed. The results are expressed as the mean ± the standard deviation (SD). Data were compared using paired Student’s *t* tests or one-way analyses of variance (ANOVAs) followed by Bonferroni tests in GraphPad Prism 8 software (San Diego, CA, USA). A *P-*value < 0.05 was considered statistically significant (^*^P<0.05; ^**^P<0.01; ^***^P<0.001).

## Results

### bmMDEs improve pancreatic islet functions in T2DM rats

bmMSCs were identified by the expression of surface markers (negative for CD45 and CD34, and positive for CD105, CD73, and CD90) (Fig. S1c), as well as by differentiation capacities toward adipocytes confirmed by Oil-Red-O staining (Fig. S1a) and toward osteoblasts confirmed by Alizarin Red staining (Fig. S1b). bmMDEs were isolated using standard differential centrifugation from cell culture supernatants. The cup-shaped membranous structure, size, and number of exosomes were identified by transmission electron microscopy (TEM) (Fig. 1a) and with a mode diameter around 100 nm via a nanoparticle tracking system (Fig. 1a, b). In addition, isolated exosomes were characterized using Western blotting to determine the presence of the established exosomal protein markers, CD9 and TSG101. Calnexin, an endoplasmic reticulum marker, was present in cells but not in exosomes (Fig. 1c). To address the biodistribution of exosomes in rats, PBS and Cy7-labeled bmMDEs were injected into each rat via the tail vein. Rats were imaged at 24 h after injections using an in vivo imaging system (IVIS) (Fig. 1d). Organs were then harvested and imaged ex vivo to clarify fluorescent signals and minimize interference (Fig. 1e).

RETRACTED

**Fig. 1:** bmMDEs ameliorate islet functions in T2DM rats. **a** Transmission electron microscopic images of bmMDEs (scale bar 50 nm). **b** Nano-sight tracking analysis was used to measure the size distribution and concentration of bmMDEs. **c** Western blotting was performed to detect protein markers (CD9, TSG101) of bmMDEs and protein markers (Calnexin) of cells. **d** Representative IVIS images of rats at 24 h after tail-vein injection with either PBS (left) or Cy7-bmMDEs (10 mg/kg, right)*.* **e** Representative IVIS images of organs (heart, lung, liver, pancreas, spleen, kidney, and gastrointestinal tract) from rats (left: PBS, right: Cy7-bmMDEs). Blood glucose after 3 h starved (**f**) and body weight (**g**) in control + PBS, T2DM + PBS, T2DM + bmMSC, and T2DM + bmMDE rats. IPGTT (**h**) and IPITT (**i**) were performed after the last intervention of bmMDEs. **j** Fasting serum insulin of control + PBS, T2DM + PBS, and T2DM + bmMDEs rats as indicated. **k** Representative sections of pancreases stained with insulin and glucagon (scale bar 20 μm). **l** The quantification of Insulin^+^ cells per islet is shown as mean ± SEM of 3 to 5 rats per group, or 4–5 pancreas sections per rat for 15–20 islets. Data are presented as the mean ± SEM (*n*=7). ^∗^*P* < 0.05, ^∗∗^*P* < 0.01, ^***^P < 0.001 (compared with the control group); ^#^*P* < 0.05, ^##^*P* < 0.01, ^###^*P* < 0.001 (compared with the T2DM group)

To evaluate the therapeutic effects of bmMDEs on T2DM, we used a rat model of T2DM based on a high-fat diet combined with STZ injections. Blood glucose was significantly reduced after bmMSC intervention (5×10^6^ cells/rat, once every 2 weeks) compared to that in the T2DM group (Fig. 1f). Additionally, bmMDEs (10 mg/kg, once every 3 days) also greatly ameliorated hyperglycemia, and blood glucose levels continued decreasing after the last infusion (Fig. 1f). Moreover, the body weight of T2DM rats was lower than that of the normal control group but was significantly increased after bmMSC or bmMDE treatment (Fig. 1g). Importantly, T2DM rats treated with bmMSCs and bmMDEs (Fig. 1h, i; Fig. S1d, e) showed significant improvement in glucose tolerance and insulin sensitivity. Serum insulin levels were dramatically decreased in the T2DM group and were elevated after bmMDE intervention compared to that in the control group (Fig. 1j). T2DM rats had a lower β-cell ratio, and the α-and-β-cell imbalance was reversed by bmMDEs (Fig. 1k, l). These data suggest that bmMDEs exerted therapeutic effects on islet function in bmMSCs in vivo.

RETRACTED

In view of the safety assessment of exosomes, previous studies have carried out relevant reports. There was no evidence that MSC-derived exosomes can cause tumorigenesis. There was no obvious hemolysis, systemic allergic reactions, and liver and kidney toxicity in different kinds of animals, and exosome infusion did not affect the body weight, liver, or kidney function of normal rats. Our results also showed that the tail-vein infusion of bmMDEs for 10 weeks had no significant effect on the liver and kidney of normal rats (Fig. S1f, g).

### bmMDEs reverse β-cell dedifferentiation in T2DM rats

Dedifferentiation caused by high glucose can lead to β-cell dysfunction [24]. We therefore investigated whether bmMDEs could alleviate the dedifferentiation level in β-cells. As shown in Fig. 2a, b and Fig. S2-1, PDX1 and FOXO1, which are markers of mature β-cells, were significantly reduced in islets of diabetic rats and were dramatically upregulated after bmMDE intervention. NGN3 and OCT4, which are markers for islet progenitor cells, were almost undetectable in islets from control rats compared with those in islets from diabetic rats. In addition, the expression levels of NGN3 and OCT4 in diabetic islets were markedly decreased after bmMDE treatment. Glucose-stimulated insulin secretion (GSIS) results showed that bmMDEs improved glucose-stimulated insulin release in diabetic islets (Fig. 2c). The mRNA levels of *Pdx1*, *Foxo1*, *Ngn3*, and *Oct4* were also consistent with the results of immunofluorescent staining (Fig. 2d).

**Fig. 2:** bmMDEs reverse β-cell dedifferentiation. **a** Paraffin-embedded sections from control + PBS, T2DM + PBS, and T2DM + bmMDE rats were immunolabeled for insulin along with mature β-cell markers (PDX1, FOXO1) and islet progenitor cells (NGN3, OCT4) (scale bar 20 μm). **b** Fluorescent-intensity expression analysis of the above indicators. **c** GSIS assays to determine insulin secretion of islets isolated from the indicated groups. RT-qPCR analyses for *Pdx1*, *Foxo1*, *Ngn3*, and *Oct4* in islets (**d**) isolated from the indicated groups. Insulin secretion in islets (**e**) of control + PBS, HG + PBS, HG + IDEs, and HG + bmMDE groups. RT-qPCR analyses for *Pdx1*, *Foxo1*, *Ngn3*, and *Oct4* in islets (**f**) from the above groups. Data are presented as the mean ± SEM (^∗^*P* < 0.05; ^∗∗^*P* < 0.01; ^***^P < 0.001)

High-glucose-induced β-cell loss commonly leads to islet dysfunction. Therefore, we investigated the effects of bmMDEs on β-cell dysfunction in primary islets and in the INS-1 cell line. First, we used mannitol (MA) as an osmotic pressure control to eliminate the effects of osmotic pressure in HG environments. The results showed that MA had no significant effect on insulin secretion or β-cell dedifferentiation in islets and INS-1 cells, while exposure to HG environment led to a significant decrease in glucose-stimulated insulin release (Fig. S2-2a–d). The expression levels of *Pdx1* and *Foxo1* were reduced after HG stimulation in islets and INS-1 cells, and the levels of *Ngn3* and *Oct4* were obviously elevated in islets but not significantly different in INS-1 cells from those in the normal control group (Fig. S2-2c, d), which indicated that HG-induced INS-1 dedifferentiation was relatively insufficient. Next, bmMDEs were labeled with PKH67 green and were co-cultured with INS-1 cells, after which cytoskeletons were visualized using incubation in rhodamine phalloidin for 24 h to detect exosomal uptake in INS-1 cells (Fig. S2-2e). GSIS results showed that bmMDEs improved the reduction of glucose-stimulated insulin release in islets (Fig. 2e) and INS-1 cells (Fig. S2-2f). Real-time quantitative PCR (RT-qPCR) analysis showed that bmMDEs could upregulate the expression of *Pdx1*, *Foxo1* in HG-induced islets and INS-1 cells, and downregulate the expression of *Ngn3* and *Oct4* in islets (Fig. 2f, Fig. S2-2g).

RETRACTED

In all of the above results, normal control exosomes (IDEs) had no effects in HG-treated islets or INS-1 cells. These data suggest that treatment with bmMDEs reversed β-cell dedifferentiation both in vivo and in vitro.

### MiR-146a in bmMDEs reverses β-cell dedifferentiation

We next explored how bmMDEs reversed dedifferentiation of β-cells. Exosomes can regulate physiological activities through exosomal miRNAs [25, 26]. We therefore conducted high-throughput sequencing of miRNA profiles in IDEs, HG-treated INS-1-cell-derived exosomes (HIDEs), and bmMDEs. A heat map was created to identify the differentially abundant miRNAs (Fig. 3a), and 10 of the most upregulated miRNAs in bmMDEs were subjected to validation by RT-qPCR. The expression levels of all 10 miRNAs in bmMDEs were higher than those in IDEs and HIDEs (Fig. 3b). We then performed a screen for the functional miRNA using the GSIS experimental setup in INS-1 cells. After pretreatment with top 10 miRNA mimics, the cells were then incubated with HG medium for 72 h. As shown in Fig. 3c, miR-146a-5p (miR-146a) mimics significantly increased insulin secretion that was otherwise inhibited by high-glucose environments compared to those of the other nine miRNA mimics. The overexpression efficiencies of miRNAs are shown in the Supporting information, namely in Fig. S3a. In addition, miR-146a mimics also ameliorated deleterious effects of HG in islets (Fig. S3b, c). RT-qPCR analysis further confirmed that treatment with bmMDEs elevated the expression level of miR-146a in both INS-1 cells and primary cultured islets (Fig. 3d, e). Furthermore, expression levels of *Pdx1* and *Foxo1* increased, while those of *Ngn3* and *Oct4* decreased in the HG + miR-146a-mimic group, compared with those in the HG + miR-NC-mimic group in primary cultured islets (Fig. 3f–i). To further investigate the role of miR-146a, INS-1 cells (Fig. S3d) and islets (Fig. S3e) were transfected with an miR-146a inhibitor. As expected, the effect of bmMDEs on islets was abolished by an miR-146a inhibitor (Fig. 3j–m). Collectively, these data demonstrate that miR-146a in bmMDEs mediated the reversal of the dedifferentiated state of β-cells.

RETRACTED

**Fig. 3:** MiR-146a in bmMDEs reverses β-cell dedifferentiation. **a** Heat map of miRNA sequencing showing the differently expressed miRNAs in IDEs, HG IDEs, and bmMDEs. **b** RT-qPCR verification of the expression levels of the top 10 differential miRNAs. **c** A GSIS assay was performed to detect insulin stimulation in HG-treated INS-1 cells transfected with the top 10 differential miRNA mimics. Levels of miR-146a in INS-1 cells (**d**) and islets (**e**) treated with bmMDEs. RT-qPCR analyses for *Pdx1*, *Foxo1*, *Ngn3*, and *Oct4* in islets (**f**–**i**) transfected with an miR-146a mimic or miR-NC mimic as indicated. mRNA expression levels of *Pdx1*, *Foxo1*, *Ngn3*, and *Oct4* in islets (**j**–**m**) transfected with an miR-146a inhibitor or miR-NC inhibitor as indicated. Data are presented as the mean ± SEM (^∗^*P* < 0.05; ^∗∗^*P* < 0.01; ^***^P < 0.001)

### Exosomal miR-146a directly targets *Numb* in β-cells

To explore the mechanism of how miR-146a regulates β-cell function, TargetScan (https://www.targetscan.org) was used to predict the potential targets of miR-146a. Among all of the predicted targets with conserved sites of miR-146a, NUMB, a human homolog membrane-bound protein [27], was noteworthy. It is known that NUMB is upregulated in diabetic patients and positively regulates the expression of NGN3, a marker of islet progenitor cells [28–30]. We found that the expression level of NUMB was significantly upregulated in islets within T2DM rats compared with that in the control group, and that bmMDE treatment decreased NUMB expression (Fig. 4a; Fig. S4a). We then confirmed that *Numb* expression was enhanced after HG treatment and was downregulated by an miR-146a mimic at the mRNA level in islets (Fig. 4b), as well as at the protein level in INS-1 cells (Fig. 4c; Fig. S4b). Subsequently, we found that bmMDEs reduced the expression of *Numb* post-HG treatment, whereas an miR-146a inhibitor attenuated this effect of bmMDEs in terms of mRNA in islets (Fig. 4d) and at the protein level in INS-1 cells (Fig. 4e; Fig. S4c). Through bioinformatic analysis, we found that the 3′UTR of the *Numb* gene contained putative binding sites for miR-146a (Fig. 4f). To further verify the association between *Numb* and miR-146a, luciferase reporter plasmids containing the wild-type 3′UTR (*Numb* 3′UTR WT) and mutated 3′UTR (*Numb* 3′UTR MUT) of *Numb* were generated. We then found that miR-146a mimics significantly reduced luciferase activity in INS-1 cells containing *Numb* 3′UTR WT but had no significant effect on *Numb* 3′UTR MUT cells (Fig. 4g). Furthermore, to determine the function of NUMB on islets, we overexpressed full-length *Numb* (Fig. S4d, e) and knocked down *Numb* expression (Fig. S4f, g) with small interfering RNAs (siRNAs) in islets. GSIS experiments showed that *Numb* overexpression reduced GSIS, and inhibition of *Numb* attenuated the inhibition of GSIS by the HG environment (Fig. 4h, m). Finally, we examined the effect of NUMB on the dedifferentiation of islet β-cells in vitro. RT-qPCR results showed that the expression levels of *Pdx1* and *Foxo1* were significantly decreased after *Numb* overexpression and that the expression levels of *Ngn3* and *Oct4* were significantly increased (Fig. 4i–l). The effect achieved after suppressing *Numb* was similar to that of miR-146a mimics shown in Fig. 3f–i (Fig. 4n–q). These data demonstrate that *Numb* is the direct downstream target of miR-146a-5p in the regulation of β-cell function and dedifferentiation.

RETRACTED

**Fig. 4:** Exosomal miR-146a directly targets *Numb* in β-cells. **a** Immunofluorescent staining for NUMB expression in pancreatic sections (scale bar 20 μm). RT-qPCR analyses of the mRNA levels of *Numb* in islets transfected with miR-146a mimics (**b**) or treated with an miR-146a inhibitor combined with bmMDEs (**d**). Western blotting for NUMB in INS-1 cells transfected with miR-146a mimics (**c**) or treated with an miR-146a inhibitor combined with bmMDEs (**e**), β-actin was used as the loading control. **f** Schematic of the sequence that miR-146a targets in the WT or mutated 3′UTR of *Numb* mRNA. **g** Luciferase activity of *Numb* WT or mutated 3′UTR reporter plasmids in INS-1 cells transfected with miR-146a mimics or miR-NC mimics as indicated. A GSIS assay was performed to detect insulin stimulation in islets transfected with *Numb* overexpression (**h**) or siRNA (**m**). RT-qPCR analyses for *Pdx1*, *Foxo1*, *Ngn3*, and *Oct4* in islets transfected with *Numb* overexpression (**i**–**l**) or siRNA (**n**–**q**). Data are presented as the mean ± SEM (^∗^*P* < 0.05; ^∗∗^*P* < 0.01; ^***^P < 0.001)

RETRACTED

### MiR-146a/*Numb* improves β-cell function through β-catenin nuclear translocation

β-catenin is a known signaling molecule that is downstream of *Numb* [31]. β-catenin has been shown to modulate pancreatic ontogenesis and islet function [32, 33]. Therefore, we explored whether β-catenin mediates the ameliorative effects of bmMDEs in our T2DM model in vitro. First, we examined the protein levels of β-catenin under different intervention conditions. We found an increase in nuclear protein levels of β-catenin in islets treated with bmMDEs, whereas the protein level of β-catenin in the cytoplasm was not changed (Fig. 5a, Fig. S5a). Similar results were examined in the miR-146a-mimic group (Fig. 5b; Fig. S5b). The effect of bmMDEs increasing the nuclear protein level of β-catenin protein was attenuated when the expression of miR-146a was inhibited (Fig. 5c; Fig. S5c). To confirm activation of the β-catenin signaling pathway, XAV-939, a β-catenin inhibitor, was used to promote β-catenin degradation. GSIS was impaired after XAV-939 intervention, and miR-146a mimics effectively attenuate this damage (Fig. 5d). We then found that miR-146a mimics elevated the expression levels of *Pdx1* and *Foxo1* and decreased expression levels of *Ngn3* and *Oct4* in HG-treated islets. However, the effect of miR-146a mimics was partially restored when combined with XAV-939 (Fig. 5e–h). Then, we verified the relationship between *Numb* and β-catenin in primary islets and INS-1 cells, respectively. The nuclear protein levels of β-catenin decreased after *Numb* overexpression, while these levels were elevated after knock down of *Numb* (Fig. 5i, j and Fig. S5d-g). These results suggest that *Numb*/β-catenin may be downstream effectors of miR-146a in the regulation of islets and β-cell function and dedifferentiation.

**Fig. 5:** MiR-146a/*Numb* reverses β-cell dedifferentiation and improves β-cell function through β-catenin nuclear translocation. **a** Nuclear translocation of β-catenin detected after bmMDE treatment in primary islets, as indicated by Western blotting analysis. **b**, **c** Western blotting for nuclear translocation of β-catenin in primary islets transfected with miR-146a mimics or treated with an miR-146a inhibitor combined with bmMDEs. Glucose-stimulated insulin secretion (**d**) in islets transfected with miR-146a mimics combined use XAV-939. **e**–**h** RT-qPCR analyses for *Pdx1*, *Foxo1*, *Ngn3*, and *Oct4* in islets transfected with miR-146a mimics combined use XAV-939. Confirmation of the changes of β-catenin nuclear translocation of *Numb* overexpression (**i**) and siRNA (**j**). β-actin and GAPDH were used as loading controls. Data are presented as the mean ± SEM (^∗^*P* < 0.05; ^∗∗^*P* < 0.01; ^***^P < 0.001)

RETRACTED

### MiR-146a knockdown abolishes bmMDE-mediated reversal of β-cell dedifferentiation in vivo

To test whether miR-146a is required for the efficacies of bmMDEs in vivo, we knocked down miR-146a expression via lentiviruses in bmMSCs (Fig. S6a). As expected, the level of miR-146a in exosomes derived from miR-146a-knockdown bmMSCs (miR-146a KD bmMDEs) was decreased significantly compared with that from exosomes derived from miR-NC-knockdown bmMSCs (miR-NC KD bmMDEs) (Fig. S6b). Exosomes were then injected into T2DM rats to detect their effects on β-cell function in vivo. Levels of blood glucose rose to ~18 mmol/L at week 5 in all rats after STZ injection. However, blood glucose of rats decreased dramatically after bmMDE intervention in the T2DM + bmMDEs^miR-NC KD^ group (~10 mmol/L at week 10), as compared with that in the T2DM + PBS group (~18 mmol/L at week 10) and T2DM + bmMDEs^miR-146a KD^ group (~16.5 mmol/L at week 10, Fig. 6a). The body weight of T2DM rats was significantly increased after bmMDEs^miR-NC KD^ treatment, but there was no statistical difference compared with that in the bmMDEs^miR-146a KD^-treated group (Fig. S6c). T2DM rats treated with bmMDEs^miR-NC KD^ showed significant improvement in glucose tolerance and insulin sensitivity, and, as expected, the effect of bmMDEs was abolished via miR-146a knockdown (Fig. 6b–e). Moreover, serum insulin levels in the T2DM + bmMDEs^miR-NC KD^ group were significantly higher than those in the T2DM + PBS group and T2DM + bmMDEs^miR-146a KD^ group (Fig. 6f). Next, immunofluorescent staining was performed in pancreatic tissue sections from bmMDE-treated rats to examine dedifferentiation of islets in vivo. The expression levels of PDX1 and FOXO1 were increased in islets, while those of NGN3 and OCT4 were decreased in T2DM rats after bmMDE^miR-NC KD^ treatments compared with those in the T2DM + PBS group and T2DM + bmMDEs^miR-146a KD^ group (Fig. 6g; Fig. S6d). RT-qPCR results of corresponding primary cultured islets demonstrated that bmMDEs upregulated the expression levels of *Pdx1* and *Foxo1* and decreased expression levels of *Ngn3* and *Oct4*, while the effects of bmMDEs were abolished by miR-146a knockdown in T2DM rats (Fig. 6h–k). These data indicate that exosomes without miR-146a attenuated their ability to improve β-cell function and reverse dedifferentiation.

**Fig. 6:** MiR-146a-knockdown bmMSC-derived exosomes fail to reverse β-cell dedifferentiation in vivo. **a** Blood glucose in control + PBS, T2DM + PBS, T2DM + bmMDE^miR-NC KD^, and T2DM + bmMDE^miR-146a KD^ rats. **b**–**e** IPGTT and IPITT were performed after the last intervention of bmMDEs^miR-NC KD^ and bmMDEs^miR-146a KD^. Values of the areas under the curve in IPGTT and IPITT were measured. **f** Fasting serum insulin of control + PBS, T2DM + PBS, T2DM + bmMDE^miR-NC KD^, and T2DM + bmMDE^miR-146a KD^ rats as indicated. **g** Paraffin-embedded sections from the indicated groups were immunolabeled for insulin along with PDX1, FOXO1, NGN3, and OCT4 (scale bar 20 μm). **h**–**k** RT-qPCR analyses for *Pdx1*, *Foxo1*, *Ngn3*, and *Oct4* in islets from the above groups. Data are presented as the mean ± SEM (^∗^*P* < 0.05; ^∗∗^*P* < 0.01; ^***^P < 0.001)

RETRACTED

## Discussion

The declining function of pancreatic β-cells is central to the progression of T2DM, and it has been confirmed that β-cell dedifferentiation is an important mechanism leading to functional β-cell reduction [5, 34, 35]. In recent years, MSC-based therapies have been demonstrated as potential approaches for treating diabetes and other diseases [36, 37]. However, some disadvantages of MSCs—such as their tumorigenic potential, issues in inducing thrombosis, and low survival times in vivo—have limited their clinical applications. Increasing evidence has suggested that exosomes, an important manifestation of paracrine actions, are the underlying substances that mediate the therapeutic effects of MSCs [38–40]. Our present results also confirmed that bmMDEs had similar therapeutic effects to those of bmMSCs on islet functions.

Hyperglycemia-induced dedifferentiation is an important mechanism that leads to β-cell failure [35, 41–43], and we found that β-cells in diabetic rats and primary islets with high glucose interventions lost their identities and turned into pancreatic endocrine progenitors that featured by high levels of *Ngn3* and *Oct4*, as well as significantly decreased expression of *Pdx1* and *Foxo1*. These results are consistent with previous reports [6, 44]. However, in the bmMDE treatment group in our present study, β-cell markers were restored and dedifferentiation markers were suppressed, indicating that bmMDEs may alleviate the dedifferentiation of β-cells. These findings suggest novel treatment effects of bmMDEs in mitigating hyperglycemia-induced β-cell dysfunction.

Exosomes regulate many physiological activities through exosomal miRNAs [37, 45]. In our present study, miR-146a emerged from our non-biased sequencing and subsequent functional screen. Interestingly, miR-146a has previously been characterized in the context of T2DM [46, 47]. For example, miR-146a is significantly lower in diabetic patients than in healthy controls and is significantly overexpressed in T2DM patients treated with metformin [48]. Liu et al. found that miR-146a mimics improve diabetic retinopathy by regulating IRAK1/TRAF6 and their downstream pro-inflammatory gene expressions [47]. Beatrix et al. discovered that miR-146 is a potential therapeutic target for the treatment of diabetic retinopathy through its inhibition of NF-κB activation [49]. Roggli et al. indicated that miR-146a was upregulated in human pancreatic islets after exposure to pro-inflammatory cytokines, and inhibition of miR-146a leads to improved β-cell function [50]. In addition, Anna et al. showed that compared with human pancreatic islets (24 h), INS-1 cells have a rapid (<6 h) expression of inflammatory genes induced by cytokine signaling, and the expression of miR-146a is downregulated upon exposure in INS1 cells after 24 h. Transfection of INS1 cells with miR-146a-5p also downregulates islet inflammation and β-cell death in part by impaired NF-κB and MAPK signaling [51]. In our study, high glucose intervention for 72 h is a chronic stimulus, and the decrease in miR-146a-5p expression may be a combination of alterations secondary to changes in the transcription of early immediate response genes and compensatory/restorative responses. However, further verification in human pancreatic islets or β-cell derived from hiPSC/hESC is still needed to make the conclusion more convincing.

RETRACTED

Next, we discussed the specific role and mechanism of miR-146a in regulating β cell dedifferentiation. After consulting the TargetScan database and previous studies, we found that the miR-146a downstream target gene, *Numb*, is upregulated in diabetic patients and positively regulates the expression of the islet progenitor cell marker, NGN3. Here, we then indicated that miR-146a negatively regulated β-cell dedifferentiation by directly binding to 3′UTR of *Numb* mRNA and inhibited its expression in β-cells. Even though the association between miR-146a and *Numb* has been reported previously [52–54], our study demonstrated, for the first time, that bmMSC-derived exosomal miR-146a rescued diabetic β-cell dysfunction via *Numb* inhibition.

β-catenin has been reported to be a downstream target gene that is negatively regulated by *Numb* and is linked to the regulation of islet function [54, 55]. To further understand the mechanism underlying *Numb*-mediated responses, we investigated β-catenin signaling in the context of diabetic β-cell dysfunction. We demonstrated that bmMDE treatments or miR-146a mimics enhanced β-catenin nuclear translocation. Moreover, miR-146a mimics rescued the inhibition of β-catenin, islet dysfunction, and dedifferentiation caused by XAV-939. We also verified the targeting relationship between Numb and β-catenin. These results highlight that the miR-146a/*Numb*/β-catenin signaling pathway is a crucial mediator of bmMDE-induced amelioration of hyperglycemia-induced β-cell dysfunction.

RETRACTED

## Conclusion

In summary, our present findings elucidate a novel mechanism by which bmMDEs regulate islet function and β-cell dedifferentiation. Results from T2DM rats and primary islets indicated that the beneficial effects of bmMDEs were mainly achieved via the miR-146a-5p/*Numb*/β-catenin pathway (Fig. 7). Our findings shed light on the potential of MSC-derived exosome-based therapeutic approaches for treating diabetes.

**Fig. 7:** Working model of bmMSC-derived exosomal miR-146a in reversing diabetic β-cell dedifferentiation. Exosomes derived from mesenchymal stem cells reverse diabetic β-cell dedifferentiation via the miR-146a/*Numb*/β-catenin signaling pathway

## Supplementary Information

**Additional file 1.**

**Additional file 2.**

**Additional file 3.**

## Data Availability

The datasets used and analyzed during the current study are available from the corresponding author on reasonable request.

## Abbreviations

MSCs: Mesenchymal stem cells
bmMSC: Bone marrow mesenchymal stem cell
bmMDEs: Bone marrow mesenchymal stem cell-derived exosomes
IDEs: INS-1-derived exosomes
T2DM: Type 2 diabetes mellitus
IPGTT: Intraperitoneal glucose tolerance test
IPITT: Intraperitoneal insulin tolerance test
AUC: Area under the curve
FBS: Fetal bovine serum
PBS: Phosphate-buffered saline
HFD: High-fat diet
HG: High glucose
MA: Mannitol
NC: Negative control
TEM: Transmission electron microscopy
GSIS: Glucose-stimulated insulin secretion
PDX1: Pancreatic duodenal homeobox-1
FOXO1: Forkhead box-containing protein O1
NGN3: Neurogenin-3
OCT4: Octamer-binding transcription factor-4
